The article "MiR-129-5p Inactivates NF-κB Pathway to Block Rheumatoid Arthritis Development via Targeting BRD4" was retracted in 2023. Reasons: signs of a paper mill; suspected computer-generated content; unreliable results or conclusions; lack of ethics approval or compliance.

# MiR-129-5p Inactivates NF-*κ*B Pathway to Block Rheumatoid Arthritis Development via Targeting BRD4

**DOI:** 10.1155/2022/8330659

**Published:** 2022-04-19

**Authors:** Zhaoli Wu, Disi Chen

**Affiliations:** ^1^Department of Integrated TCM & Western Medicine, Hunan Provincial People's Hospital, Changsha 410005, Hunan, China; ^2^Department of Respiratory Medicine, Hunan Provincial People's Hospital, Changsha 410005, Hunan, China

## Abstract

**Methods:**

The abundance of miR-129-5p was detected in the samples including normal tissues and RA tissues and cell lines including human fibroblast-like synoviocytes (hFLSs) and human rheumatoid arthritis fibroblast-like synoviocytes (RA-FLSs). The CCK-8 assay, flow cytometry, Transwell, and ELISA were used to observe the effects of miR-129-5p on the phenotype of RA-FLSs. Moreover, the potential targets of miR-129-5p were identified with TargetScan and dual-luciferase reporter gene assay. Besides, the abundances of the proteins were analyzed with western blot.

**Results:**

Decreased miR-129-5p was observed in RA tissues and cells. Increased miR-129-5p obviously blocked the proliferation, inflammatory stress, and migration and remarkably promoted cellular apoptosis. Moreover, BRD4 was confirmed as targets of miR-129-5p, and BRD4 upregulation could partly rescue the inhibition of miR-129-5p on aggressive behaviors of RA-FLSs. Besides, the finding of this study also proved that upregulated miR-129-5p could impede the NF-*κ*B pathway via targeting BRD4.

**Conclusion:**

This study suggests that miR-129-5p suppresses the activation of NF-*κ*B pathway to block the progression of RA via targeting BRD4.

## 1. Introduction

Rheumatoid arthritis (RA) is still an intractable disease with high incidence in middle-aged and senior people. The patients with RA always exhibit persistent inflammatory reactions in synovial tissue, neovascularization, and joint destruction. Moreover, persistent inflammation may also induce multiple severe complications such as lung and cardiovascular disease [1, 2]. The aggressive behaviors of RA fibroblast-like synoviocytes (RA-FLS) are direct reason causing RA development. RA-FLSs are characterized with the high aggressive behaviors including high proliferative and migratory abilities [3, 4]. Moreover, the matrix metalloproteinases (MMPs) produced by RA-FLSs can promote the joint injury which may cause irreversible joint dysfunction for the patients [5]. Therefore, the intervention of suppressing the aggressive phenotype of RA-FLSs has been suggested as a promising strategy for RA treatment in clinical.

The disorder of microRNA profile acts as a biomarker event for RA progression [6]. Moreover, accumulating reports have indicated that miRNAs directly regulate RA development via influencing the proliferation, inflammatory level, and cellular molecular signal transduction of RA-FLSs [7, 8]. MiR-129-5p, located on p13, functions as a tumor obstructor to restrain malignant behaviors of cancer cells. MiR-129-5p plays a critical role in bone development, and miR-129-5p has been confirmed to promoter the differentiation of bone marrow mesenchymal stem cells [9]. Moreover, several reports have indicated that aberrant abundance of miR-129-5p is associated with multiple bone diseases. The research has revealed that miR-129-5p is associated with osteoarthritis development [10]. Moreover, the study has also found that miR-129-5p downregulation may promote the progression of RA [11]. However, the research studies on regulation mechanism of miR-129-5p in RA are still necessary.

The article "MiR-129-5p Inactivates NF-κB Pathway to Block Rheumatoid Arthritis Development via Targeting BRD4" was retracted in 2023. Reasons: signs of a paper mill; suspected computer-generated content; unreliable results or conclusions; lack of ethics approval or compliance.

This study was aimed to investigate the functions and molecular mechanism of miR-129-5p in RA development.

## 2. Materials and Methods

### 2.1. Sample Collection

The specimens including RA and normal tissues were stored at −70°C. This experiment has been approved by the Hospital Ethics Committee.

### 2.2. Cell Culture and Transfection

The human rheumatoid arthritis fibroblast-like synoviocytes (RA-FLSs) were purchased from Beijing Donggeboye Biotechnology Co., Ltd (Beijing, China). The cell medium was DMEM supplying 10% FBS and 1% penicillin/streptomycin. The cells were cultured in the conditions including 37°C and 5% CO_2_. Moreover, the cell subculture was performed when cell density was at 90%.

For cell transfection, 4 g of DNA (or 100 pmol RNA) and 10 *μ*l Lipofectamine 2000 were mixed with 250 *μ*l medium and incubated for 5 min, respectively. Subsequently, the medium containing DNA (or RNA) was mixed and incubated with the medium containing Lipofectamine 2000 for 20 min at 25°C. Finally, 500 *μ*l of mixture was added into each well, and then cells were incubated for 24 h.

### 2.3. qRT-PCR

RA-FLSs were treated with TRIzol reagent for RNA extraction, and the related concentration was measured with spectrophotometry. Subsequently, PrimeScript® RT reagent Kit (Thermo Fisher, Massachusetts, USA) was applied for cDNA reverse transcription. Briefly, 10 *μ*L of the reaction system for qRT-PCR was performed with following conditions: for miRNA, 95°C for 5 min followed by 40 cycles of 95°C for 15 s and 60°C for 1 min; for mRNA, 95°C for 5 min, followed by 40 cycles of 95°C for 15 s, 62°C for 30 s, and 72°C for 30 s. The abundance of the related miRNA or mRNA was calculated with 2^−(ΔΔCt)^. The primers of the genes are listed in Table 1.

### 2.4. Western Blotting

The abundance of the proteins in RA-FLSs was observed by western blot. In brief, the cells were treated with the RIPA buffer for 30 min on the ice, and then total proteins were extracted from the cells with centrifugation (13,200 rpm for 15 min). The BCA kit was applied for concentration measurement of proteins. The proteins, mixed with loading buffer, were boiled for 5 min. The proteins were separated with SDS-PAGE and then translated on PVDF membranes. The membranes were incubated with the primary antibodies (anti-BED4, ab243862 abcam; anti-P65, ab32536, abcam) at 4°C overnight after immersing in 5% fat-free milk for 2 h. TBST was used to wash membranes for three times, and second antibodies were used for membrane incubation at 25°C for 2 h. Finally, the abundance of the proteins was observed by a chemiluminescence detection system after removing redundant second antibodies by TBST.

The article "MiR-129-5p Inactivates NF-κB Pathway to Block Rheumatoid Arthritis Development via Targeting BRD4" was retracted in 2023. Reasons: signs of a paper mill; suspected computer-generated content; unreliable results or conclusions; lack of ethics approval or compliance.

### 2.5. Flow Cytometry

2 × 10^3^ cells RA-FLSs were suspended with 200 *μ*L ice Annexin V-FITC binding buffer. Subsequently, 10 µL of propidium iodide (PI 20 µg/ml) and 5 µl of Annexin V-FITC (10 µg/ml) were used for cell staining in the dark for 5 min. The apoptosis of the cells was detected with a flow cytometry equipment (BD Biosciences, State of New Jersey, USA).

### 2.6. CCK-8 Assay

5 × 10^3^ cells were seeded into 96-well plates. After transfection for 24 h, 48 h, 72 h, and 96 h, the cells were added with 10 *μ*L of CCK-8 solution and then incubated for 4 h under lightless condition. Finally, the OD450 value of the cells was detected with microplate reader.

### 2.7. Dual-Luciferase Report Genes Assay

The sequences of BRD4 wild type (BRD4-wt) and BRD4 mutant type (BRD4-mut) with mutant sites in the binding region with miR-129-5p were inserted into pmirGLO vector (Youbao Biotechnology Co., Ltd, Chongqing, China), respectively. After that, miR-NC/miR-129-5p mimics and BRD4-wt/BRD4-mut were used for the transfection of RA-FLSs. Finally, after culturing for 48 h, the luciferase activity in the cells was measured.

### 2.8. Transwell Assay

2 × 10^4^ cells were cultured in upper chamber of Transwell plates to normal growth stage. After transfection for 72 h, the cells were cultured with 200 *μ*L serum-free medium, and 500 *μ*L DMEM plus 10% FBS was supplied into lower chamber. The cells were cultured at 37°C for 24 h and then were fixed with formaldehyde for 30 min. Subsequently, the cells in upper chamber were removed with a cotton ball. Finally, the migratory cells were calculated in 3 randomly visual regions.

### 2.9. ELISA

The ELISA kits (Shanghai Fusheng Biotechnology Co., Ltd, Shanghai, China) were applied for the detection of inflammatory factors including IL-6 and IL-1*β*. The detection process was performed following the instructions of the kits, strictly.

The article "MiR-129-5p Inactivates NF-κB Pathway to Block Rheumatoid Arthritis Development via Targeting BRD4" was retracted in 2023. Reasons: signs of a paper mill; suspected computer-generated content; unreliable results or conclusions; lack of ethics approval or compliance.

### 2.10. Data Analysis

The experiments were repeated for 3 times, independently. SPSS 20.0 was applied for data analysis, and the difference of the data was judged with Chi-squared test or ANOVA with Tukey's post hoc-test. Moreover, Graphpad Prism 8 was used for data visualization.

## 3. Results

### 3.1. Decreased miR-129-5p Was Observed in RA-FLSs

To investigate the connection of miR-129-5p and RA development, the abundance of miR-129-5p was detected in RA tissues and cells. The results revealed that miR-129-5p was remarkably upregulated in the RA samples (Figure 1(a); *P* < 0.01). Besides, compared with the human fibroblast-like synoviocytes (hFLSs), decreased miR-129-5p was observed in the RA-FLSs (Figure 1(b); *P* < 0.01). Those evidences hinted that miR-129-5p upregulation was involved in the progression of RA.

### 3.2. Increased miR-129-5p Suppressed the Aggressive Behaviors of RA-FLSs

To illustrate the functions of miR-129-5p in RA-FLSs, miR-129-5p was upregulated in RA-FLSs to observe the changes in phenotype of RA-FLSs. The results proved that miR-129-5p upregulation effectively suppressed the proliferation and migration and induced the apoptosis of RA-FLSs (Figures 2(a), 2(c), and 2(d); *P* < 0.01). Moreover, miR-129-5p downregulation also effectively improved the inflammatory levels in RA-FLSs (Figure 2(b); *P* < 0.01). Those proofs suggested that miR-129-5p can inhibit the inflammatory apoptosis of RA-FLSs.

### 3.3. BRD4 Was Directly Regulated by miR-129-5p

To reveal the regulation mechanism of miR-129-5p in RA, miRDB and TargetScan database were used to screen the downstream factors of miR-129-5p. The prediction result showed that miR-129-5p could directly bind with BRD4. Moreover, the luciferase reporter gene assay also confirmed that miR-129-5p mimics reduced luciferase activity of RA-FLSs transfected with the wt-BRD4 (Figure 3(a); *P* < 0.01). Moreover, reduced BRD4 was also found in the RA-FLSs compared with that in normal FLSs (Figure 3(b); *P* < 0.01). Those observations supported that BRD4 was directly regulated by miR-129-5p.

### 3.4. BRD4 Reversed the Effects of miR-129-5p on RA-FLSs

To verify whether miR-129-5p can inhibit the progression of RA via regulating BRD4, the expressed vectors of miR-129-5p and BRD4 were used for RA-FLSs transfection to observe the changes in phenotype of RA-FLSs. The results showed that suppressed proliferation, invasion, and inflammatory responses induced by increased miR-129-5p were reversed by BRD4 upregulation (Figures 4(a)–4(d); *P* < 0.01). Those observations hinted that miR-129-5p affected the behaviors of RA-FLSs via inhibiting BRD4.

The article "MiR-129-5p Inactivates NF-κB Pathway to Block Rheumatoid Arthritis Development via Targeting BRD4" was retracted in 2023. Reasons: signs of a paper mill; suspected computer-generated content; unreliable results or conclusions; lack of ethics approval or compliance.

### 3.5. MiR-129-5p Inactivated the NF-*κ*B Pathway via Suppressing BRD4

To delve the molecular mechanism of miR-129-5p in RA development, the activity of NF-*κ*B pathway was analyzed in RA-FLSs after transfecting with the expressed vectors of miR-129-5p and BRD4. The results confirmed that increased miR-129-5p distinctly reduced the abundances of BRD4, P65, and p-P65 (Figure 5; *P* < 0.01). In addition, BRD4 upregulation partly rescued the inactivation of miR-129-5p on NF-*κ*B pathway (Figure 5; *P* < 0.01).

## 4. Discussion

RA is still a spiny question for modern medical therapeutic system and may induce irreversible motor dysfunctions of the patients [12]. Considerable research studies have proved that the aggressive behaviors of RA-FLSs are direct reason causing the persistent pathological changes in joints [13, 14]. Disorder miRNA profile has been found as a biomarker event in RA-FLSs [15]. This study investigated the connection of miR-129-5p with RA, revealed the functions and regulation of miR-129-5p on the aggressive behaviors of RA-FLSs, and provided some references for the RA treatment.

Accumulating research studies have indicated that abnormal miRNA profile is a distinguishing feature of RA, and some miRNAs have been confirmed to involve the development of this disease [16]. In this study, decreased miR-129-5p was observed in RA-FLSs compared with normal cells. MiR-129-5p serves as an intruder role to impede the formation and development of multiple diseases. The research has confirmed that miR-129-5p is obviously reduced in the tissues of the patients with osteoarthritis, and miR-129-5p upregulation could remarkably improve the IL-1*β*-mediated osteoarthritis via suppressing HMGB1 [17]. Moreover, miR-129-5p has been confirmed to block the proliferation and induce the apoptosis of RA-FLSs via directly regulating the expression of IGF-1 [11]. The finding of this study also proved that miR-129-5p functioned as a suppressor to inhibit the proliferation and invasion of RA-FLSs. MiR-129-5p has been verified to involve the release of inflammatory factors, and increased miR-129-5p can effectively alleviate the levels of inflammatory response in multiple diseases including acute kidney and intestinal injury [18, 19]. The observation in this study also confirmed that increased miR-129-5p could effectively relief the IL-6 and IL-8 levels. Thus, it suggests that miR-129-5p plays an inhibitor role in progression of RA.

MiRNAs are characterized with restraining the translation process to influence the phenotype of cells via interacting with the related mRNAs. For RA, the miRNAs also serve as important regulators in the pathological changes of the cells. The study has indicated that miR-130a reduces the proliferation and inflammation of RA-FLSs via targeting NDRG2 [20]. Wang et al. have discovered that miR-129-5p functions as a inhibitor role in multiple myeloma, and increased miR-129-5p could restrain multiple malignant behaviors of tumor cells via targeting JAG1 [21]. The major observation in this research was that miR-129-5p was involved in RA development via directly targeting BRD4. BRD4 upregulations have been found in multiple diseases. For bone disease, increased BRD4 also mediates the inflammatory reactions and aberrant proliferation of cells [21]. BRD4 has been confirmed as a promising therapeutic target for osteoarthritis, and decreased BRD4 could effectively improve the inflammatory stress in osteoarthritis [22]. Moreover, this study also confirmed that BRD4 could effectively reverse the effects of miR-129-5p on RA-FLSs.

The article "MiR-129-5p Inactivates NF-κB Pathway to Block Rheumatoid Arthritis Development via Targeting BRD4" was retracted in 2023. Reasons: signs of a paper mill; suspected computer-generated content; unreliable results or conclusions; lack of ethics approval or compliance.

RA development is related with the dysfunctions of multiple cellular pathways including JAK/STAT, PI3K/AKT, NF-*κ*B, and so on. Crispino et al. have indicated the abnormally activated JAK/STAT pathway in RA-FLSs, and the inhibition of JAK/STAT pathway can effectively alleviate the pain and symptoms of the patients with RA [23]. This study also observed the aberrant activation of NF-*κ*B pathway in RA-FLSs. Several reports have indicated that activated NF-*κ*B pathway is involved in promoting the multiple aggressive behaviors of RA-FLSs, such as excessive proliferation and violent invasion [24]. Inactivating NF-*κ*B pathway has been considered as a promising strategy for restraining the RA development. This study confirmed that increased miR-129-5p could effectively reduce the activity of NF-*κ*B pathway. MiR-129-5p has been confirmed to take part in attenuating the lipopolysaccharide-mediated acute kidney injury via regulating the activity of NF-*κ*B pathway [18]. Moreover, it was also found that miR-129-5p inactivated NF-*κ*B pathway in RA-FLSs was related with BRD4. For RA, several research studies have also proved that BRD4 upregulation is critical reason for NF-*κ*B pathway which may promote the progression of this arthropathy [25]. For osteoarthritis, decreased BRD4 could reduce the activity of NF-*κ*B and thus block the progression of the disease. The study has also indicated that BRD4 can inhibit the ubiquitination of RelA to increase the stability of NF-*κ*B [26]. Therefore, it implies that miR-129-5p regulates the activity of NF-*κ*B pathways via targeting BRD4.

## 5. Conclusion

In summary, this study suggests that miR-129-5p could regulate the activity of NF-*κ*B pathways to block the aggressive behaviors of RA-FLSs by targeting BRD4.

The article "MiR-129-5p Inactivates NF-κB Pathway to Block Rheumatoid Arthritis Development via Targeting BRD4" was retracted in 2023. Reasons: signs of a paper mill; suspected computer-generated content; unreliable results or conclusions; lack of ethics approval or compliance.

## Figures and Tables

**Figure 1:** The related abundance of miR-129-5p in RA tissues and cells. (a) Normal tissues vs. RA tissues. (b) hFLSs vs. RA-FLSs. ^*∗∗*^*P* < 0.01.

**Figure 2:** MiR-129-5p effectively suppressed the aggressive behaviors of RA-FLSs. (a) Cell viability detected by CCK-8 assay. (b) Inflammatory factor levels detected by ELISA. (c) Cell migration observed by Transwell. (d) Cell apoptosis detected by flow cytometry assay. ^*∗∗*^*P* < 0.01.

**Figure 3:** BRD4 was a downstream target of miR-129-5p. (a) Dual-luciferase report gene assay. (b) The mRNA abundance of BRD4. ^*∗∗*^*P* < 0.01.

**Figure 4:** MiR-129-5p effectively suppressed the aggressive behaviors of RA-FLSs via targeting BRD4. (a) The viability of RA-FLSs observed by CCK-8 assay. (b) Inflammatory factor levels detected by ELISA. (c) Cell migration observed by Transwell. (d) Cell apoptosis detected by flow cytometry assay. ^*∗∗*^*P* < 0.01.

**Figure 5:** MiR-129-5p inhibited NF-*κ*B pathway via targeting BRD4. (a) The related abundance of miR-129-5p. (b–e) The abundances of BRD4, P65, and p-P65 measured with western blot. ^*∗∗*^*P* < 0.01.

**Table 1:** Primer sequence of genes.

miR-129-5p-F	5'-: ACCCAGTGCGATTTGT-3'
miR-129-5p-R	5'-: ACTGTACTGGAAGATGGA-3'
BRD4-F	5'-ACAACAAGCCTGGAGATGACA-3'
BRD4-R	5'-GTTTGGTACCGTGGAAACGC-3'
U6-F	5'-CTCGCTTCGGCAGCACA-3'
U6-R	5'-AACGCTTCACGAATTTGCGT-3'

## Data Availability

The data used to support the findings of this study are available on reasonable request from the corresponding author.
